# Hysterectomy by Transvaginal Natural Orifice Transluminal Endoscopic Surgery versus Transumbilical Laparoscopic Single-Site Surgery: A Single-Center Experience from East China

This article has been retracted.

**DOI:** 10.1155/2022/8246761

**Published:** 2022-08-08

**Authors:** Bin Yan, Hui-Xian Miao, You Wang, Jia-Mu Xu, Xiu-Qing Lu, Wan-Hong He, Wen Di, Wei-Hua Lou

**Affiliations:** ^1^Department of Obstetrics and Gynaecology, Renji Hospital, School of Medicine, Shanghai Jiao Tong University, Shanghai, China; ^2^Shanghai Key Laboratory of Gynaecologic Oncology, Shanghai, China; ^3^State Key Laboratory of Oncogenes and Related Genes, Shanghai Cancer Institute, Renji Hospital, School of Medicine, Shanghai Jiao Tong University, China; ^4^Jiangsu Province Hospital, The First Affiliated Hospital with Nanjing Medical University, China

## Abstract

**Objective:**

To compare hysterectomy by transvaginal natural orifice transluminal endoscopic surgery (VNOTES) versus transumbilical laparoscopic single-site surgery (LESS) as a minimal invasive technique. *Materials and Method*. The women undergoing hysterectomy for benign diseases by VNOTES and LESS from January 2020 to June 2021 in a tertiary hospital in Shanghai were retrospectively analyzed.

**Results:**

361 women were included in our study, with 228 in the VNOTES groups, 129 in the LESS groups, and 4 conversions from VNOTES to LESS technique. The length of a VNOTES hysterectomy was shorter than that of LESS (80.76 min versus 112.09 min; MD -31.34 min; 95% CI -40.24 to -22.43 min; *P* < 0.001). VNOTES hysterectomy has a quicker gas passage by the anus (18.80 versus 36.49 hours, MD -17.68 hours, 95% CI -20.23 to -15.14 hours, *P* < 0.001) and associated with a shorter length of hospital stay (2.31 versus 3.77 days, MD -1.46 days, 95% CI -1.75 to -1.17 days, *P* < 0.001), while with no increase in blood loss during the operation (median 50 versus 50 ml, *P* = 0.25). Besides, the VAS pain score in the 24^th^ hour after the operation was lower (median 0 versus 0.5, *P* < 0.001) in the VNOTES group. Four unique phases of the learning curve were identified using cumulative analysis: the mean operation time of phase I was 82.81 ± 31.45 min (the initial learning curve of 43 cases), phase II was 72.48 ± 23.66 min (the acquisition of command of 91 cases), phase III was 103.77 ± 45.69 min (the further learning of 26 cases), and phase IV was 73.18 ± 26.89 min (postlearning in 68 cases).

**Conclusions:**

VNOTES is noninferior to LESS as a new minimal invasive procedure for hysterectomy, which also allows patients a faster recovery from surgery and to suffer less pain, and its efficiency and feasibility in large uterine need further exploring.

## 1. Introduction

Hysterectomy is one of the most common gynecological procedures for benign gynecological diseases and some early-stage tumors, such as abnormal uterine bleeding, adenomyosis, atypical endometrial hyperplasia, and cervical hyperplasia. The procedure has been performed in different ways: abdominal hysterectomy (AH), conventional vaginal hysterectomy (VH), laparoscopic hysterectomy (LH), and robotically assisted hysterectomy (RH). According to the number of laparoscope, LH can be classified into several types: conventional multiport laparoscopic hysterectomy (CMLH), laparoscopy-assisted vaginal hysterectomy (LAVH), or transumbilical laparoscopic single-site surgery (LESS). As a Cochrane review involving 5012 women reports, VH is superior to LH and AH because of its faster return to normal activities. When VH is not feasible, LH is preferred but related to more urinary tract injuries [1]. Although patients appear to benefit more from VH, it is not easy to have a good command of VH because of its poor visualization and limited space for manipulation.

Recently, natural orifice transluminal endoscopic surgery (NOTES), which utilizes the natural orifices such as the rectum, mouth, urethra, and vagina to get into the peritoneal cavity, has been developed since its minimal invasions during procedures. After various animal experiments, NOTES started to be used in human and the first transvaginal NOTES (VNOTES) hysterectomy was performed in 2012 [2]. VNOTES is a combination of conventional vaginal surgery and laparoscopic single-site surgery, which overcomes the limitations of conventional VH with the help of endoscopic view and instruments. Several studies have reported VNOTES as a safe procedure, associated with shorter surgical time, faster postoperative recovery, reduced postoperative pain, decreased postoperative wound infections, and cosmetic results [3, 4].

LESS is reported as a feasible, safe, and equally effective alternative to CMPL for hysterectomy [5]. A randomised controlled trial of VNOTES has suggested that VNOTES is noninferior to CMPL for hysterectomy and reduces postoperative pain [6, 7]. Our study was aimed at comparing VNOTES with LESS as a minimally invasive technique for hysterectomy. We explored that VNOTES, as a combination of VH and LESS, not only removes the uterus as safely and effectively as LESS but has a faster recovery from the procedure and better cosmesis. What is more, we evaluated the learning curve of the new technique, evaluating its efficiency and feasibility in uterine with normal weight. Learning curve means the learning time or times required for new technologies or methods.

## 2. Materials and Method

This was a retrospective study of women who underwent hysterectomy by transvaginal NOTES and by LESS with the same indications from January 2020 to June 2021 in Shanghai Jiao Tong University affiliated Renji Hospital, a teaching hospital in China. The surgical indications include atypical endometrial hyperplasia, adenomyosis, uterine myoma, high-grade cervical dysplasia, treatment-refractory dysfunctional uterine bleeding, benign adnexal masses, and uterine prolapse. The following information was collected in all the patients: age, body mass index (BMI), prior vaginal birth, previous abdominal surgery, diabetes, cardiovascular diseases, indication for operation, uterine weight, total operation time, intraoperative and postoperative complications, and the length of hospital stay.

The duration of the operation was defined as the time from the start of circumcising the vaginal mucosa to the removal of the uterus. The VAS pain score was accomplished in the first 24 hours after the operation. The complications were accepted as wound infection, blood transfusion requirement, and readmission into the hospital in 6 weeks.

The learning curve of the VNOTES technique was measured as the operation time over the time course of the study. Cumulative sum (CUSUM_OT_) analysis was used as reported by previous studies [8, 9]. The CUSUM calculated the total difference between the individual values and mean of all values. Arranging the patients in sequence, graphical information of the trend in the operation time of consecutive procedures could be plotted. The CUSUM_OT_ for the 1st case was the difference between the OT for the 1st case and the mean OT for all patients. The CUSUM_OT_ of the 2nd case was the CUSUM_OT_ of the 1st value added to the difference between the OT of the 2nd case and the mean OT for all patients. The calculation was repeated until the last CUSUM_OT_ reached zero. Linear regression with log transformations was performed to determine the sign of the slope of regression.

### 2.1. Surgical Procedure

All participants in our study were admitted into hospital several days earlier (depending on the severity of the complications) to receive the laboratory and imaging assessment to rule out the contraindications of the surgery, especially those who could not tolerate the surgery. The operations were performed by the same expert gynecologist (Lou), who was the first gynecologist to conduct the VNOTES procedures in our department. All women in our study received hysterectomy and either bilateral salpingectomy or salpingo-oophorectomy depending on the indications. The first step of the hysterectomy was to circumcise the vaginal mucosa around the cervix by using a scalpel, then expose the vesical peritoneal reflection after pushing up the anterior vaginal mucosa along the uterine cervical fascia, and dissect the peritoneal reflection to get access to the abdominal cavity anteriorly. Similarly, the posterior vaginal wall was exposed and dissected, and the pouch of Douglas was opened. The uterosacral ligament complexes were then cut as done in the conventional vaginal surgeries, followed by circumcising the cervix to get into the peritoneal cavity. To achieve a pneumoperitoneum, a VNOTES port (Beijing Hang Tian KaDi Technology R&D Institute) was inserted through the vagina into the peritoneal cavity, which had two 5 mm and two 10 mm channels. The two endoscopic instruments were used through the two 5 mm channels and a standard 10 mm rigid mm 30° laparoscope (Stryker) through one 10 mm channel. As done in the conventional vaginal surgery, the hysterectomy was performed caudally to cranially. The bilateral ureters would routinely be identified during the operation but not be dissected unless it was necessary. The uterine vessels and bilateral ligaments, including parametrial tissues, round ligament, ovarian proper ligament, and mesosalpinx, were cut and sealed by the ultrasonic scalpel and the endoscopic instrument with bipolar coagulation (Hangzhou Kangji Medical Instrument). When the salpingo-oophorectomy was indicated, the bilateral infundibulopelvic ligaments would also be cut to enable the ovaries to be disconnected. The free uterine was removed through the vagina. After confirming there was no active bleeding, the VNOTES port was removed and the vaginal cuff was closed using one 1-0 suture (Ethicon Endo-Surgery, Norderstedt, Germany) through the vagina.

In those who received hysterectomy by LESS, the gynecologist performed hysterectomy by transumbilical laparoscopic single-site surgery technique. A LESS port was inserted through the umbilicus to create access to the abdominal cavity, which also had two 5 mm and two 10 mm channels. A standard 10 mm rigid 30° laparoscope (Stryker) and endoscopic instruments were used. Similarly, the ureters were identified but not dissected to prevent injuries. With the help of a uterine manipulator and endoscopic instruments with bipolar coagulation, the gynecologist performed hysterectomy cranially to caudally. The uterine was removed through the vagina, which in some extent would save surgical time. The vaginal cuff was also closed using the 1-0 suture (Ethicon Endo-Surgery, Norderstedt, Germany). The umbilicus was closed using absorbable suture after ensuring there was no bleeding inside the abdominal cavity. Finally, a wound dressing was used on the umbilicus.

### 2.2. Statistical Analysis

The Fisher exact test or chi-square test was applied for dichotomous secondary outcome measures, while an independent *t*-test or Mann–Whitney *U* test was applied for the continuous secondary outcomes. *P* values of <0.05 were considered to indicate statistical significance. Data analysis was performed by using SPSS software (version 26).

## 3. Results

Between January 2020 and June 2021, a total number of 232 patients received hysterectomy by VNOTES and 129 by LESS. Four cases in the VNOTES group failed to remove the uterus and converted to LESS technique, which resulted in a conversion rate of 1.72% (*P* = 0.30). The 4 conversions were all diagnosed as multiple uterine myoma, 3 of whom failed due to the large size of myoma (up to 12 centimeters) and 1 of whom due to the adhesion between the uterus and the pelvis.

Baseline characteristics were comparable between the two groups except for some certain surgical indications, which are summarized in Table 1. The percentage of uterine myoma and benign adnexal tumor in the VNOTES group was lower than that in the LESS group (36.84% versus 48.44%, *P* = 0.04, and 4.82% versus 20.16%, *P* < 0.001), while the percentage of cervical dysplasia and uterine prolapse was higher than that in the controlled group (29.82% versus 14.07%, *P* < 0.001, and 4.82% versus 0.78%, *P* < 0.02).

As shown in Table 2, we leave out the 4 conversions and compared the main outcomes between the two groups. In our study, not only the median uterine weight was comparable between the VNOTES group and the LESS group (median 164.00 gram versus 176.90 gram, *P* = 0.58) but also the percentage of uterine weight more than 400 g (*P* = 0.48) was comparable. The total length of a VNOTES hysterectomy was shorter than a LESS one (78.21 minutes versus 112.09 minutes; mean difference (MD) -33.89 minutes; 95% confidence index (CI) -42.55 to -25.22 minutes; *P* < 0.001). Compared with LESS hysterectomy, VNOTES hysterectomy has a quicker gas passage by the anus (18.80 versus 36.49 hours, MD -17.68 hours, 95% CI -20.23 to -15.14 hours, *P* < 0.001) and thus associated with a shorter length of hospital stay (2.31 versus 3.77 days, MD -1.46 days, 95% CI -1.75 to -1.17 days, *P* < 0.001). Surprisingly, the VNOTES and LESS groups shared a similar blood loss during the operation (median 50 versus 50 ml, *U* = 2662.5, *z* = −1.152, *P* = 0.25, there was no statistical difference; a Mann–Whitney *U* test).

The VAS pain score in the 24th hour after the operation in the VNOTES group was lower than that in the LESS group (median 0 versus 0.5, *U* = 2133.0, *Z* = −3.517, *P* < 0.001, there was statistical difference; a Mann–Whitney *U* test). The less analgesic use in the VNOTES group also indicated patients suffered less pain from VNOTES technology (odds ratio 4.00, 95% CI 1.81 to 8.84, *P* < 0.001). There was exudation in the umbilicus wound in 2 women in the LESS group; however, it showed no statistical difference (*P* = 0.13). Besides, no complications and readmission in 6 weeks were reported in both groups.

Then, after getting the raw operation time in each consecutive patient in chronological order (Figure 1), we calculated the CUSUM_OT_ values and a learning curve was achieved, which was plotted in a graph as shown in Figure 2(a). The learning curve was able to be divided into four distinct phases: cases 1-43 into the initial learning phase (phase I), cases 44-134 into the commanding phase (phase II), cases 135-150 into the further learning phase (phase III), and cases 150-228 into postlearning phase (phase IV). The best fit curves of the learning curve in each phase are shown in Figure 2(b).

There were significant differences among the four phases in operation time and uterine weight (Table 3). Patients in phase III had the longest operation time (103.77 ± 45.69 min) and the largest uteri (423.27 ± 338.14 grams, Figures 3(a) and 3(b)) but shared similar BMI and postoperative stay with the other three phases.

## 4. Discussion

Since the VNOTES was introduced into our department in 2019, more and more patients preferred this advanced technique to receive hysterectomy. In our study, we retrospectively analyzed the cases of hysterectomy by VNOTES and LESS, involving as much as 228 patients in the VNOTES group. We found that VNOTES was noninferior to LESS hysterectomy and could be an alternative for hysterectomy in women with benign diseases due to its minimal invasiveness, as previously reported [10–12]. In our study, with no increased risk of blood loss during the procedure, VNOTES had a shorter surgical length compared with the LESS group, which saved almost half an hour, though part of which might resulted from the leave out of suturing the umbilical wound. There were no increase in the intra- and postoperative complications in the VNOTES group, which also proved VNOTES was a safe technique for hysterectomy. Besides, women in the VNOTES group had a faster recovery with less pain from the surgery. Women after the VNOTES surgery had a faster recovery of gastrointestinal function and thus had a reduced length of hospital stay, which no doubt decreased the hospitalization expenses. We investigated the VAS pain score in the 24th hour after the surgery and postoperative analgesic use, which suggested women in the VNOTES group suffered less postoperative pain. No postoperative and wound infection was reported after the procedure. Further, VNOTES had an outstanding cosmetic result since it created no apparent wound. Most patients in the VNOTES group expressed their satisfaction of this technique when they were followed up in the outpatient clinic. In summary, VNOTES provided a more minimal invasive procedure for women to undergo hysterectomy.

Four cases in the VNOTES groups were converted to the LESS technique. Large uterine size is reported to have a significant effect on operative time and blood loss [13, 14], and the prior intra-abdominal procedures might contribute to adhesions, which would be challenging to successfully perform the hysterectomy especially for VNOTES and thus increased blood loss and operative time [15, 16], which was corresponding to our findings. We assumed our 4 failures may be contributed to the position of the fibroid and the pelvic adhesion. In one case, a 12-centimeter fibroid grew into right broad ligament and grew caudally to the cervix, which resulted in obstruction in the route to the abdominal cavity. In another case, who had a prior abdominal surgery, it was not easy to separate the vesical peritoneal reflection because of the firm adhesion and therefore caused a failure of entrance into the abdominal cavity.

Due to its feasibility and applicability, we evaluated the learning curve of the VNOTES technique. In phase I, which was the initial stage, it took 43 cases to acquire the basic skill in completing VNOTES with or without adnexectomy. In phase II, the phase of commanding the technique, 91 cases were needed to solidate the technique. In our study, the surgeon practiced 134 cases to fully master the new technique. Therefore, in phase III, the surgeon built up the confidence and tried to perform the surgery in more challenging cases, in which uterine weight was much heavier than the other three phases and two failures happened during this phase. An increasing operation time and blood loss were seen in this phase. This indicated that VNOTES for large uterine might not be so efficient for uterine weight of around 430 g or less. In phase IV, the postlearning phase, the surgeon had achieved proficiency in uterine with normal weight and showed a good command of the technique. In our study, we suggested that increasing operation time might be associated with heavier uterine weight, which implied it of great importance to evaluate the uterine volume before the surgery.

Inevitably, our study had several limitations. Our study was a single-center trial in one teaching hospital and all the operations were performed by one expert gynecologist, which might result in limitations in the generality of some findings. A multicenter trial involving more gynecologists needs to be conducted to reconfirm the findings. LESS was proved to achieve a lower pain score faster than CMPL [17]. In 1989, laparoscopic technique was introduced into this operation, which changed the surgical approach and concept of hysterectomy [18]. A lot of changes have taken place in laparoscopic technique. In our study, we evaluated the postoperative pain score. Further study could be conducted to find out if the VNOTES group could achieve a lower pain score faster than LESS and whether it could be equally efficient in large uterine.

## 5. Conclusion

VNOTES, a combination of VH and LESS, could be a new minimal invasive procedure for hysterectomy. VNOTES allows patients to have a faster recovery from surgery and to suffer less pain. In the future, a randomised comparison between VNOTES and VH could be done to assess the effectiveness of both techniques.

## Figures and Tables

**Figure 1:** Raw operation time (OT) of 228 patients in a chronological order.

**Figure 2:** (a) The CUSUM_OT_ values of operation time in four phases. (b) The best fit curve for each phase.

**Figure 3:** (a) Graph of raw uterine weight plotted against a chronological case number (228 consecutive patients). (b) The average uterine weight in four phases.

**Table 1:** Baseline characteristics of the population.

	VNOTES^∗^ (*n* = 228)	LESS (*n* = 129)	*P* value
Age (years)	53.04 ± 9.44	54.26 ± 10.33	0.27
BMI (kg/m^2^) (range)	23.96 ± 3.08	24.26 ± 3.84	0.48
Prior vaginal birth, *n*(%)	155 (67.98)	80 (62.02)	0.25
Previous abdominal surgery, *n* (%)	84 (36.84)	59 (45.74)	0.10
Cardiovascular disease, *n* (%)	41 (17.98)	32 (24.81)	0.13
Diabetes, *n* (%)	13 (5.70)	5 (3.88)	0.45
Indication for surgery, *n* (%)			
Atypical endometrial hyperplasia	16 (7.02)	5 (3.91)	0.23
Adenomyosis	36 (15.79)	13 (10.16)	0.13
Uterine myoma	84 (36.84)	62 (48.44)	0.04
Cervical dysplasia	68 (29.82)	18 (14.07)	<0.001
Treatment-resistant DUB	2 (0.88)	4 (3.13)	0.20
Benign adnexal tumor	11 (4.82)	26 (20.16)	<0.001
Uterine prolapse	11 (4.82)	1 (0.78)	0.02

DUB: dysfunctional uterine bleeding; SD: standard deviation. ^∗^The 4 conversions were not included.

**Table 2:** Main outcomes in the population.

	VNOTES (*n* = 228)	LESS (*n* = 129)	*P* value
Uterine weight (g), median (±IQR)	164.00 (±224.00)	176.90 (±254.00)	0.58
Uterine weight > 400 g, *n*(%)	31 (13.6)	21 (16.3)	0.48
Total operating time (min), mean (±SD)	78.21 ± 30.79	112.09 ± 44.05	<0.001
Blood loss (ml), median (±IQR)	50 (±10)	50 (±50)	0.25
Duration of anal exhaust (hours) (±SD)	18.80 ± 6.60	36.49 ± 13.71	<0.001
VAS pain score, mean (±IQR)	0 (0-0)	0.5 (0-5)	<0.001
Hospital stay (d), median (±IQR)	2.31 ± 0.69	3.77 ± 1.57	<0.001
Postoperative analgesics use, *n* (%)	10 (4.39)	20 (15.50)	<0.001
Complications, *n*(%)	0 (0)	0 (0)	—
Wound infection, *n*(%)	0 (0)	2 (1.55)	0.13
Readmission after 6 weeks, *n*(%)	0 (0)	0 (0)	—

**Table 3:** Interphase comparison of patient characteristics and postoperative outcomes.

	Phase I (*n* = 43, cases 1-43)	Phase II (*n* = 91, cases 44-134)	Phase III (*n* = 26, cases 135-160)	Phase IV (*n* = 68, cases 161-228)	*P*
BMI (kg/m^2^)	24.01 ± 2.74	24.32 ± 3.46	22.57 ± 2.27	24.06 ± 2.93	0.09
Uterine weight (g)	158.92 ± 134.60	195.96 ± 154.25	423.27 ± 338.14	214.30 ± 171.89	<0.001
Operation time (min)	82.81 ± 31.45	72.48 ± 23.66	103.77 ± 45.69	73.18 ± 26.89	<0.001
Blood loss (ml)	50.00 ± 30	50.00 ± 20	50.00 ± 113	50.00 ± 18	0.01^∗^
Postoperative stay (days)	2.23 ± 0.43	2.52 ± 0.94	2.20 ± 0.41	2.14 ± 0.43	0.12

^∗^There was significant difference between phases I, II, III, and phase IV.

## Data Availability

The datasets used and analyzed during the current study are available from the corresponding author on reasonable request.
